# Co-occurrence of problematic facebook and video game use: prevalence and association with mental health disorders among adolescents

**DOI:** 10.1186/s40359-024-01842-2

**Published:** 2024-07-02

**Authors:** Sihem Ben Fredj, Mohamed Ouertani, Nawel Zammit, Rim Ghammam, Jihen Maatoug, Firas Chouikha, Imed Harrabi, Hassen Ghannem

**Affiliations:** 1 Faculty of Medicine of Sousse, University of Sousse, Sousse, 4000 Tunisia; 2 Department of Epidemiology, Farhat Hached University Hospital, “LR19SP03”, Sousse, 4000 Tunisia

**Keywords:** Problematic Facebook use, Problematic video game use, Risk factors, Adolescent, Mental health

## Abstract

**Introduction:**

The rapid proliferation of technology and its impact on adolescents’ lives have raised concerns about addictive behaviors and its potential consequences, including behavioral and mental health problems. This study investigates the prevalence and risk factors associated with the co-occurrence of Problematic Facebook Use and Problematic Video game Use among Tunisian adolescents.

**Methodology:**

We conducted a cross-sectional study in the urban area of Sousse governorate in Tunisia during the 2018/2019 school year. We selected a representative sample of high school students enrolled in public educational institutions in Sousse. Data collection was performed through a self-administered structured questionnaire, which gathered information on sociodemographic characteristics, lifestyle behaviors, and mental health disorders. Problematic Facebook Use was assessed using the validated Arabic version of the Bergen Scale, while Problematic Video Game Use was measured using the 21-point Lemmens Scale, which was translated into Arabic. Statistical analysis was carried out using the SPSS program (version 20).

**Results:**

We enrolled a total of 1342 high school students in our study, of whom, 63.2% were female with a mean age of 17.5 ± 1.44 years. The prevalence of Problematic Facebook Use and Problematic Video Game Use was  28.3% and  13% respectively. Regarding the co-occurrence of the two problematic behaviors, 31.3% of participants faced a singular addictive behavior, either related to problematic Facebook or video game use, while 5% had both addictive behaviors simultaneously. In a multivariate analysis, risk factors for the co-occurrence of Problematic Facebook and Video Game Use, in decreasing order of significance, included severe depression (AOR = 4.527; *p* = 0.003), anxiety (AOR = 4.216; *p* = 0.001), male gender (AOR = 4.130; *p* < 0.001), problematic internet use (AOR = 3.477; *p* = 0.006), as well as moderate depression (AOR = 3.048; *p* = 0.007).

**Conclusion:**

Our study found that Problematic Facebook and Video Game Use were prevalent among Tunisian adolescents. The co-occurrence of these disorders is strongly linked to male gender, problematic internet use, depression, and anxiety disorders. These findings underscore the urgency of implementing tailored and effective awareness and prevention programs to address these emerging challenges.

**Supplementary Information:**

The online version contains supplementary material available at 10.1186/s40359-024-01842-2.

## Introduction

Over the past few decades, the rapid emergence of new technologies, such as laptops, smartphones, and the internet, has significantly enhanced various aspects of people’s lives, including their professional and educational endeavors [1]. These technologies have not only provided easy access to entertainment like video games and popular social platforms like Facebook but have also brought about potential negative consequences, especially among adolescents who are particularly vulnerable to these risks [2]. Adolescence is a crucial phase that connects childhood and adulthood, characterized by notable physiological, physical, and emotional transformations. It begins around 10–11 years for girls and 12–13 years for boys and typically lasts until approximately 24 years of age [3]. During this period, adolescents assert their individuality and explore different paths to shape their identity leading them to engage in risky behaviors like addiction [4]. Psychiatrist Aviel Goodman defines addiction as a repetitive behavior that brings pleasure and relief, despite adverse consequences and loss of control [5]. Addiction is not limited to substance abuse but also includes excessive fixation on certain screen practices and digital media like watching videos, gaming, and socializing [6–8]. Video games have gained immense popularity worldwide, with approximately 1.46 billion video game users in 2019 [9]. In addition, Facebook is globally the most widely used social media platform worldwide and boasts approximately 3 billion monthly active users [10]. The excessive use of Facebook and Video games may lead to addiction due to the elevation of dopamine levels coupled with the vulnerable traits of personality in adolescents [11, 12]. Accordingly, the rising issues of Problematic Facebook Use and Problematic Video game Use are becoming a global concern, especially among adolescents [13–20]. The fourth regional report of the Mediterranean School Survey Project on Alcohol and Other Drugs (MedSPAD) in 2022 revealed that the prevalence of school adolescents spending daily over 6 h on social media and 5 or more hours on video games during non-school days was higher in Eastern Mediterranean countries like Tunisia than Western Mediterranean countries like France, Italy, and Spain [21]. Similarly, a national Tunisian survey conducted in 2021 found that 30.1% of school adolescents spend 4 or more hours daily on social media, and a quarter devote the same amount of time to video games, with a higher proportion among boys [22]. Adolescents within Low-Middle Income Countries including Tunisia might be more susceptible to Problematic Social Media Use and Problematic Video Game Use than in High-Income Countries as a consequence of several risk factors, including economic hardships and inadequate social support [23].

Furthermore, addictive behaviors do not always occur in isolation, they frequently co-occur in the same individual, meaning that those who are addicted to one behavior tend to be addicted to several other behaviors or substances at the same time [24]. Moreover, while the literature extensively addresses elevated instances of concurrent addictive behaviors, the majority of these studies concentrate primarily on co-occurring substance-related issues, and there exists a limited body of research that delves into co-occurring technology addictions [16]. This co-occurrence of addictive behaviors exposes individuals to even greater negative consequences mainly behavioral problems (i.e. exposure to junk food marketing and sedentary lifestyles leading to weight gain and dental problems, impact body image, cyberbullying, sleep disturbances, eye problems and early exposure to explicit content, etc.) [25], and mental health problems (i.e. depression, anxiety, suicidal thoughts, etc.) [26].

Recognizing the influence of societal context on mental health aspects, there emerges a compelling need for a more comprehensive exploration of contributing factors within diverse settings [23]. Considering these reflections, our study has been undertaken to determine the prevalence and risk factors associated with the co-occurrence of Problematic Facebook and Video Game Use among adolescents enrolled in secondary schools within a Tunisian eastern region.

## Methods

### Study design

This is an analytical cross-sectional study conducted from November 2018 to January 2019 within public secondary schools, located in the city of Sousse, in eastern Tunisia.

### Study population

The target population for this study comprises all adolescents aged 15 to 18 years living in the governorate of Sousse. Meanwhile, the source population includes all adolescents aged 15 to 18 years who are currently enrolled in public educational institutions within the governorate of Sousse. The sample size was determined based on the prevalence of Problematic Facebook Use. The formula used for sample size calculation was n = ( p-q) Zα² /i², with the following parameters: a prevalence (p) of 28% for Problematic Facebook Use [27], where q = 1 - p, a significance level (α) of 5%, and a precision level (i) set at 4%. The two-stage proportional cluster sampling technique with a cluster effect of 2 was applied. To account for possible losses and unequal distribution of students across classes, a 20% contingency was added. This resulted in an estimated minimum sample size of 1162 adolescents. We made a two-stage proportional sampling approach with a cluster selection strategy to ensure a representative sample for our study. In the first stage, the city of Sousse was divided into three geographical areas: Sousse-Medina, Sousse-Jawhara, and Sousse-Riadh. One or more high schools were then selected from each area based on the density of the student population: Sousse-Medina (1 high school), Sousse-Jawhara (6 high schools), and Sousse-Riadh (3 high schools). We included a total of four high schools out of the ten eligible high schools (with a number of students > 500) using simple random sampling.

In the second stage, we stratified the classes by grade level (1st, 2nd, 3rd, or 4th grade) and by teaching section (mathematics, experimental sciences, economics, computer science, technical, or literary section). From a total of 144 classes across the four high schools, we randomly selected 59 classes in proportion to the number of classes at each academic level. The distribution of selected classes was as follows:14 classes out of 35 classes within 1st grade, 12 classes out of 32 classes within 2nd grade, 15 classes out of 33 classes within 3rd grade, and 18 classes out of 44 classes within 4th grade.

All students present in the randomly drawn classes who expressed willingness to participate and obtained consent from their legal guardians were included in the study. A total of 1342 students from these selected classes were invited to participate in the study.

### Data collection

The data collection period extended from November 2018 to January 2019. Before starting data collection, we obtained approval from the Regional Directorate of Education in Sousse, as well as the consent of the directors and teachers at the selected high schools. The data collection sessions were held in the classrooms of high school students and lasted approximately one hour on average. Before administering the survey, a trained research team introduced the study’s objectives. We also reassured the students about the confidentiality and anonymity of their responses. Following the introduction and their consent to participate, students completed self-administered questionnaires in their respective classrooms during regular class sessions. The researchers vocalized each question allowing students to respond before proceeding to the next question. This method ensured the completeness and integrity of collected data.

### Measures

Data were collected using a structured self-administered and pretested questionnaire written in literary Arabic [28]. The questionnaire consists of three sections *(i) Socio-demographic characteristics*: This section includes questions about age, gender, academic level, study section, year of repetition, parents’ occupation and education level, and average weekly spending money; *(ii) Lifestyle behaviors*: This section aims to assess different risk behaviors among Tunisian adolescents. Physical activity was evaluated through the question, “Do you engage in at least 60 minutes of physical activity per day for five or more days per week?” with possible answers being yes or no. The average daily time spent on the internet was measured by asking participants to report their average time in hours and/or minutes. Spending more than two hours per day on Internet was considered Problematic Internet Use. Weekly pocket money was evaluated by asking students about their average weekly spending in Tunisian Dinars (TND). Tobacco experimentation was assessed by the question, “Have you ever smoked a cigarette or tried smoking at least once in your life?“, with possible answers being yes or no. Alcohol drinking was evaluated through a simple yes or no question, “Do you drink alcoholic beverages (beer, wine, whiskey, or similar)?” Experimentation with various illicit substances was assessed by asking, “Have you used one or more of these substances at least once in your life?“, with multiple-choice answers provided for various illicit substances such as cannabis, inhalants, Trihexyphenidyl, Cocaine, Heroin, Ecstasy, Subutex, Diethyllysergamide, Ketamine, Fentanyl, and others; *(iii) The Mental Health* section encompasses several vital components: self-esteem, depression, anxiety, alexithymia, Problematic Video Game Use, and Problematic Facebook Use. To measure these constructs, self-report scales were utilized, accompanied by clear and concise written instructions placed at the beginning of each questionnaire. This approach aims to ensure participants’ comprehension of the scales and their purpose, facilitating accurate and reliable responses. In addition to the instructions, a brief explanation of each construct is provided, aiding respondents in understanding the specific aspects being assessed. This meticulous methodology strengthens the validity of the data collected and contributes to the overall rigor of the study.

The Rosenberg Self-Esteem Scale (RSE) comprises two factors. The “positive self-esteem” including items 1, 2, 4, 6, and 7, assesses satisfaction with oneself, recognition of good qualities, sense of equality with others, feeling of usefulness, and maintaining a positive attitude. The “negative self-esteem,” including items 3, 5, 8, 9, and 10, explores feelings of inadequacy, lack of pride, tendencies towards self-disrespect, worthlessness, and perceived failure [29]. Respondents rate items on a four-point scale, reversed for certain items. Each factor’s score ranges from 10 to 40, with higher scores indicating greater self-esteem. A score below 25 suggests very low self-esteem, a score between 25 and 31 indicates low self-esteem, a score between 31 and 34 signifies average self-esteem, a score between 34 and 39 reflects strong self-esteem, and a score above 39 indicates very strong self-esteem [29]. The scale showed high reliabilities with a Cronbach’s alpha of 0.94.

The Beck Depression Inventory (BDI) is a widely used screening tool to measure depression severity in adults and adolescents aged 13 and above [30]. We used the shorter version with 13 items has comparable internal consistency to the original 20-item version [31]. The inventory uses a Likert scale, with items rated from 0 to 3 points, assessing a range of depression-related symptoms and attitudes, including depressed mood, pessimism, feelings of failure, lack of satisfaction, guilt, self-hatred, self-mutilation, social withdrawal, indecision, distorted body image, difficulty working, fatigue, and loss of appetite. BDI scores range from 0 to 39. Scores between 0 and 3 indicate no or minimal depression. Scores between 4 and 7 suggest mild depression, between 8 and 15 indicate moderate depression, and between 16 and 39 are indicative of severe depression.

The Arabic version of the Screen for Child Anxiety Related Disorders-Child version (SCARED-C) scale was used for the assessment of anxiety [32, 33]. The SCARED-C consists of five subscales, targeting different dimensions of anxiety counting panic disorder, generalized anxiety, separation anxiety, social phobia, and school phobia. It comprises 41 questions. Respondents rate each item on a scale of 0 (rarely), 1 (sometimes), and 2 (often). Consequently, the total score on the SCARED-C can range from 0 to 82, indicating the overall level of anxiety experienced by the child. A total score of ≥ 25 is indicative of a possible anxiety disorder. For items 1, 6, 9, 12, 15, 18, 19, 22, 24, 27, 30, and 34, a score of ≥ 7 may suggest the presence of panic disorder. A score of ≥ 9 on items 5, 7, 14, 21, 23, 28, 33, and 35 may point to generalized anxiety disorder. Similarly, a score of ≥ 5 on items 4, 8, 13, 16, 20, 25, 29, and 31 may indicate separation anxiety. Social phobia may be indicated by a score of ≥ 8 on items 3, 10, 26, 32, 39, 40, and 41. Lastly, a score of ≥ 3 on items 2, 11, 17, and 36 suggests the possibility of school avoidance.

To assess alexithymia, we used the Arabic version of the Toronto Alexithymia Scale (TAS-20) [34] The TAS-20 consists of 20 self-report items, each rated on a five-point Likert scale, and three subscales. The first, “Difficulty identifying feelings,” assesses in seven items [1, 3, 6, 7, 9, 13, 14] the ability to differentiate emotions from somatic sensations [35, 36]. The second, “Difficulty describing feelings,” evaluates in five items [2, 4, 11, 12, 17] the verbal articulation of emotions. The third, “Subscale of Outwardly Oriented Thinking,” gauges in eight items [5, 8, 10, 15, 16, 18–20] outward-focused thinking. The total alexithymia score is calculated by summing responses across items. A score ≤ 50 categorizes no alexithymia, 51–60 suggest possible alexithymia, and scores ≥ 61 indicate the presence of alexithymia.

Problematic Facebook use was assessed using the Arabic version of the Bergen Scale [37]. The Bergen Scale delves into six key dimensions, namely concentration, mood swings, tolerance, withdrawal, conflict, and relapse, with respondents providing ratings on a 5-point Likert scale (1 = very rarely, 2 = rarely, 3 = sometimes, 4 = often, 5 = very often). The total score on this scale ranges from 6 to 30, with higher scores indicating a greater degree of dependence on Facebook. For the identification of Problematic Facebook Use, the criterion used is a score of ≥ 3 on at least four out of the six items.

The Lemmens scale measures Problematic Video Game Use. The video games included were those played on computers, consoles, smartphones, or tablets. It evaluates seven dimensions of addiction, including significance, tolerance, mood modification, relapse, withdrawal, conflict, and problems, each represented by three items. Respondents rate these items on a 5-point Likert scale. Problematic Video Game Use is defined as a score of 9 or higher on at least four out of seven dimensions, indicating consistent engagement in problematic gaming behaviors. In our study, the scale was translated into Arabic through a rigorous process involving bilingual researchers and experts to maintain clarity and original meaning. The scale showed high reliabilities with a Cronbach’s alpha of 0.94.

### Statistical analysis

The statistical analyses were conducted using the Statistical Package for Social Sciences (SPSS version 20) for Windows. Qualitative variables were summarized using absolute and relative numbers and percentages. For quantitative variables, means and standard deviations were reported if the data followed a normal distribution. We examined the co-occurrence of Problematic Facebook Use and Problematic Video Game Use based on ratios of observed and expected prevalence. The expected proportion was calculated by multiplying the individual probabilities of each risk factor based on their occurrence in the study population. The difference between the observed and the expected proportion (O/E) was calculated. If the result of the ratio of observed-to-expected (O/E) is greater than 1, it indicates the existence of aggregation between the Problematic Facebook and Video Game Use. To assess the factors associated with the co-occurrence of these problematic behaviors, we conducted a Chi-square test. Subsequently, a multivariate analysis was carried out using multinomial logistic regression, following the stepwise top-down strategy. All explanatory variables that demonstrated a significance level of < 0.2 in the univariate analysis were included in the initial multivariate analysis models. The final models presented the results of the factors associated with the dependent variable, expressed as adjusted Odds ratios (ORs) along with their corresponding 95% confidence intervals (95% CIs). For all tests conducted, the statistical significance level was defined as 5%.

### Ethical considerations

The study obtained ethical approval from the Farhat Hached University Hospital’s ethics committee and consent from the Regional Directorate of Education. High-school directors and teachers were informed about the study beforehand. Informed consent was acquired from parents and legally authorized representatives of students, who also provided their consent. Measures were taken to protect data confidentiality, with no personal identifiers used. We maintain participant privacy during data collection, ensuring anonymity and security. Data were processed within the epidemiology department, with restricted access.

## Results

### General characteristics of the study population

The study encompassed a cohort of 1342 high school students, with a notable majority of 63.2% identifying as female, yielding a sex ratio of 1.72. The average age of the participants stood at 17.5 ± 1.44 years. Within this group, 45% fell within the age bracket of 16 to 18 years, while 17.3% were situated between 14 and 16 years, and the remaining 37.7% were above 18 years of age. In terms of educational paths, 25.8% of participants pursued a general academic curriculum (1st year of secondary level), and 27.6% opted for experimental sciences. Approximately 28.1% of students acknowledged repeating a class at some point. As for the educational background of parents, 41.7% of fathers and 37.5% of mothers possessed a university degree. Regarding parental occupation, 26.3% of fathers were engaged in independent professions, while 46.9% of mothers identified as housewives. The median weekly allowance received by the students was 10 Tunisian Dinars (TD), with an Inter-Quartile Range spanning from 5 to 20 TD. For a comprehensive overview of the sociodemographic characteristics of the entire participant cohort, refer to Table 1.

**Table 1:** Summary table of socio-demographic characteristics of Tunisian adolescents (*n* = 1342)

Socio-demographic characteristics	*n*	%
Gender		
Male	494	36.8
Female	848	63.2
Age		
[14–16]	232	17.3
[16–18]	604	45.0
> 18	506	37.7
School level		
1st year	344	25.8
2nd year	287	21.4
3rd year	354	26.2
4th year	357	26.6
History of repeating a year		
Yes	374	28.1
No	959	71.9
Father’s level of education		
Illiterate	27	2.0
Primary	181	13.6
Secondary	444	33.4
University	555	41.7
Don’t know	123	9.3
Mother’s level of education		
Illiterate	57	4.3
Primary	215	16.2
Secondary	463	34.8
University	498	37.5
Don’t know	96	7.2
Profession of the Father		
No occupation	26	2.0
Blue-collar worker	221	16.9
Free profession	344	26.3
Public servant	306	23.4
managerial employee	250	19.1
Other	160	12.3
Mother’s occupation		
No occupation	621	46.9
Blue-collar worker	123	9.3
Free profession	105	7.9
Public servant	312	23.5
managerial employee	124	9.4
Other	40	3.0
Weekly pocket money		
≤ 10 TND	743	59.4
> 10 TND	507	40.6

N: number; %: prevalence

### Lifestyle habits and mental health

The prevalence of Problematic Facebook Use and Problematic Video Game Use among adolescents was 28.3% and 13% respectively. A notable proportion of adolescents (66.8%) manifested signs of alexithymia. Furthermore, 11.4% of the participants presented severe depression. Likewise, 39% of students experienced low or very low levels of self-esteem. More than half of the participants (67%) demonstrated symptoms of anxiety disorders. Problematic Internet use was observed in 72.4% of adolescents. Physical inactivity was reported in 57.6% of cases. In terms of smoking behavior, 27% of the adolescents acknowledged having smoked at least once in their lifetime. As for current cigarette use, 10.3% of the participants reported smoking at least one cigarette in the previous month. Current water pipe use was revealed in 6.6% of the participants, while electronic cigarette was used by 11.1% of adolescents. nearly, 6% of the adolescents acknowledged using alcohol. Moreover, 9% of the adolescents experimented with illicit substances at least once in their lifetime (Table 2).

**Table 2:** Results of lifestyle habits and the mental health assessment among Tunisian adolescents (*n* = 1342)

Column1	*n*	%
**Problematic Video Game Use**	157	13.0
**Problematic Facebook Use**	345	28.3
**Alexithymia**		
No alexithymia	187	13.9
Possible Alexithymia	259	19.3
Alexithymia	896	66.8
**Depression**		
No depression	465	34.6
Mild depression	303	22.6
Moderate depression	421	31.4
Severe depression	153	11.4
**Self-esteem**		
Very low or low	508	39.0
Within the average	489	37.6
Strong or very strong	305	23.4
**Anxiety disorder**	899	67.0
Panic disorder	817	60.9
Generalized anxiety disorder	649	48.4
Separation Anxiety	750	55.9
Social phobia	536	39.9
School avoidance	520	38.7
**Recommended physical activity**	555	42.4
**Problematic Internet Use**	972	72.4
**Tobacco experimentation**	358	27.0
**Consumption of alcohol**	79	6.1
**Experimentation with inhalants and illicit substances**	120	9.0

N: number; %: prevalence

### Co-occurrence of problematic facebook and video game use

Most adolescents (64%) had 0 addictive behaviors for Facebook and video games, while only 5% had both Problematic Facebook and Video Game Use. The proportion of students with a combination of problematic behaviors was higher than would be expected based on individual frequencies (O/A ratio = 1.3) (Table 3).

**Table 3:** Prevalence of the cooccurrence of problematic facebook and video game use among Tunisian adolescents (*n* = 1342)

				Prevalence	
Number of problematic behaviors	Problematic Facebook Use	Problematic Video Game Use	Observed *n* (%)	Expected *n* (%)	O/E
**0**	─	─	699 (63.7)	686 (62.5)	1
**1**	**+**	─	246 (22.4)	259 (23.6)	0.9
	─	**+**	97 (08.9)	110 (10.0)	0.9
**2**	**+**	**+**	55 (05.0)	42 (03.9)	1.3

O/A: Observed/Expected

### Risk factors for the co-occurrence of problematic facebook and video game use

In terms of univariate analysis, the prevalence of the co-occurrence of Problematic Facebook and Video Game Use was significantly higher among adolescents who repeated at least one grade than those without a history of repeating years (7.8% versus 4%, *p* < 0.001), adolescents whose mothers were illiterate or had a primary level education than those who reported that their mothers had a secondary and a university level of education (6.9% versus 4.8% and 3.7% respectively), and those whose fathers were illiterate or had a primary level education than those who reported that their fathers had a secondary and a university level of education (9.2% versus 5% and 3.7% respectively) (Table 4).

**Table 4:** Association of the co-occurrence of problematic facebook and video game use with sociodemographic characteristics among Tunisian adolescents (*n* = 1342)

	0	1	2	
	*n* (%)	*n* (%)	*n* (%)	*p*
**Gender**				0.097
Boys	249(63.4)	117(29.7)	27(06.9)	
Girls	450(63.9)	226(32.1)	28(04.0)	
**Age**				**0.402**
[14–16]	130(68.8)	48(25.4)	11(05.8)	
]16–18]	309(62.9)	160(32.6)	22(04.5)	
> 18	260(62.4)	135(32.4)	22(05.3)	
**Level of education**				**0.712**
1st year	172(61.9)	89(32.0)	17(06.1)	
2nd year	150(61.7)	78(32.1)	15(06.2)	
3rd year	184(64.6)	88(30.9)	13(04.6)	
4th year	193(66.3)	88(30.2)	10(03.4)	
**History of repeating years**				**< 0.001**
Yes	165(53.4)	120(38.8)	24(07.8)	
No	530(67.9)	220(28.2)	31(04.0)	
**Mother’s level of education**				**0.004**
Illiterate or primary level	122(56.2)	80(36.9)	15(06.9)	
Secondary level	247(63.0)	126(32.1)	19(04.8)	
University level	292(71.2)	103(25.1)	15(03.7)	
**Father’s level of education**				**0.001**
Illiterate or primary level	97(55.7)	61(35.1)	16(09.2)	
Secondary level	225(62.0)	120(33.1)	18(05.0)	
University level	324(70.9)	116(25.4)	17(03.7)	
**Weekly pocket money**				**0.407**
≤ 10 TND	377(62.1)	200(32.9)	30(04.9)	
> 10 TND	322(65.7)	143(29.2)	25(05.1)	

N: number; %: prevalence; p: significance level

0: No addictive behavior, 1: Problematic Facebook Use or Problematic Video Game Use, 2: Problematic Facebook and Video Game Use

In addition, the prevalence of the co-occurrence of Problematic Facebook and Video Game Use increased significantly (*p* < 0.001) with the studied mental health disorders such as depression, anxiety, low self-esteem, and alexithymia (Table 5). There was a statistically significant relationship between the increasing number of addictions among participants and problematic internet use (*p* < 0.001) and tobacco experimentation (*p* = 0.002) (Table 5).

**Table 5:** Association of the co-occurrence of problematic facebook and video game use with lifestyle habits and mental health problems among Tunisian adolescents (*n* = 1342)

	0	1	2	
	*n* (%)	*n* (%)	*n* (%)	*p*
**Self-esteem**				< 0.001
Very low or low	227(55.4)	155(37.8)	28(06.8)	
Average	264(65.0)	120(29.6)	22(05.4)	
Strong or very strong	193(74.5)	61(23.6)	5(01.9)	
**Depression**				**< 0.001**
No depression	280(74.8)	84(22.5)	10(02.7)	
Mild depression	167(66.8)	77(30.8)	6(02.4)	
Moderate depression	197(57.1)	120(34.8)	28(08.1)	
Severe depression	55(43.0)	62(48.4)	11(08.6)	
**Alexithymia**				**< 0.001**
No alexithymia	116(74.4)	37(23.7)	3(01.9)	
Possible Alexithymia	157(74.1)	46(21.7)	9(04.2)	
Alexithymia	426(58.4)	260(35.7)	43(05.9)	
**Anxiety disorder**				**< 0.001**
Yes	424(58.1)	259(35.5)	47(06.4)	
No	275(74.9)	84(22.9)	8(02.2)	
**Recommended physical activity**				**0.833**
Yes	297(64.7)	138(30.1)	24(05.2)	
No	395(63.5)	197(31.7)	30(04.8)	
**Problematic use of the Internet**				**< 0.001**
Yes	460(57.9)	286(36.0)	49(06.1)	
No	239(79.1)	57(18.9)	6(02.0)	
**Tobacco experimentation**				**0.002**
Yes	171(57.8)	100(33.8)	25(08.4)	
No	527(66.2)	239(30.0)	30(03.8)	
**Consumption of alcohol**				**0.401**
Yes	50(54.3)	36(39.1)	6(06.5)	
No	649(64.6)	307(30.5)	49(04.9)	
**Experimentation with inhalants and illicit substances**				**0.050**
Yes	58(58.0)	32(32.0)	10(10.0)	
No	638(64.3)	309(31.1)	45(04.5)	

N: number; %: prevalence; p: significance level

0: No addictive behavior, 1: Problematic Facebook Use or Problematic Video Game Use, 2: Problematic Facebook and Video Game Use

The results of the multinomial regression analysis are presented in Table 6 using the 0-addictive behavior problem category as the baseline. These results showed that boys were more likely than girls to have at least one addictive behavior (AOR = 1.475, CI_95%_ [1.070–2.034], *p* = 0.018) and the two addictive behaviors (AOR = 4.13, CI_95%_ [2.209–7.719], *p* < 0.001). Adolescents in the non-science sections were 1.398 times more likely to have an addictive behavior than those in the science sections (AOR = 1.398; CI_95%_ [1.057–1.848]; *p* = 0.019). Adolescents with problematic Internet use had a 2.327-fold increased risk of developing an addictive behavior compared to those without problematic Internet use (AOR = 2.237; CI_95%_ [1.602–3.124]; *p* < 0.001), and this risk was greater when comparing the two addictive behaviors group to the no addictive behavior group (AOR = 3.477; CI_95%_ [1.438–8.406]; *p* = 0.006). Having an anxiety disorder increased 1.707-fold the likelihood of developing at least one addictive behavior (AOR = 1.707; CI_95%_ [1.200–2.430]; *p* = 0.003) and with 4.216-fold the likelihood of developing both addictive behaviors (AOR = 4.126; CI_95%_ [1.775–10.014]; *p* = 0.001) compared to those without. In addition, adolescents with severe depression were 2.931 times more likely to have at least one addictive behavior than those without depression (AOR = 2.931; CI_95%_ [1.817–4.729]; *p* < 0.001), this risk increased with the number of addictive behaviors (OR = 4.527; CI_95%_ [1.682–12.190]; *p* = 0.003).

**Table 6:** Multinomial logistic regression (0 addictive behavior is the reference category) of the problematic facebook and video game use cooccurrence among Tunisian adolescents (*n* = 1342)

		1			2		
		AOR	CI_95%_	*p*	AOR	CI_95%_	*p*
**Gender**	Boys/Girls	**2.475**	1.070–2.034	**0.018**	**4.130**	2.209–7.719	**< 0.001**
**Problematic Internet Use**	Yes/No	**2.237**	1.602–3.124	**< 0.001**	**3.477**	1.438–8.406	**0.006**
**Anxiety**	Yes/No	**1.707**	1.200–2.430	**0.003**	**4.216**	1.775–9.559	**0.001**
**Depression**	Severe depression/No depression	**2.931**	1.817–4.729	**< 0.001**	**4.527**	1.682–12.190	**0.003**
	Moderate depression/No depression	**1.642**	1.138–2.371	**0.008**	**3.048**	1.362–6.822	**0.007**
	Mild depression/No depression	1.460	0.994–2.144	0.054	0.983	0.392–2.848	0.975

AOR: adjusted odds ratio; CI_95%_: 95% confidence interval; p: significance level

1: Problematic Facebook Use or Problematic Video Game Use, 2: Problematic Facebook and Video Game Use

## Discussion

Our study was designed among Tunisian adolescents enrolled in high schools in the city of Sousse to determine the prevalence of addictive behavior related to video games and Facebook, as well as their cooccurrences and related risk factors of this cooccurrence. Of the total of 1342 high school students selected in the final sample, the prevalence of Problematic Video Game Use was 13% and the prevalence of Problematic Facebook Use was 28.3%. Even though a significant proportion of the global youth population resides in Low-Middle Income Countries, the body of research addressing mental health and dependence disorders in these countries remains limited in comparison with High-Income Countries [2]. Limited Maghreb country research exists on this topic. Our findings aligned with previous Tunisian studies reporting 28% of Problematic Facebook Use [38] and 14% of Problematic Video Game Use [39]. Our result was higher than the prevalence estimates in North America and Western/Northern Europe, but quite lower than the prevalence estimates in Asia, Africa, and the Middle East [17].

As per recent research findings, there exists a tendency for addictive behavior to co-occur, suggesting that the likelihood of experiencing concurrently multiple addictive behaviors for different kinds of technologies is a noteworthy phenomenon [40]. This emphasizes the intricate nature of the interconnections among diverse forms of addictive behaviors [41]. However, there is a scarcity of research that explores the realm of co-occurring technological addictions [16]. In our study, three distinct groups were formed based on the number of observed addictive behaviors. The majority, accounting for 63.7% of the study population, had neither Problematic Facebook Use nor Problematic Video Game Use. About 31.3% had one addictive behavior, and 5% had two addictive behaviors. Andreassen et al. found a positive association between the addictive use of social networks and video games, and the two addictive technological behaviors shared common risk factors demonstrating the disposition of co-occurrence [42]. However, there are distinctive non-shared risk factors, such as gender. Research consistently indicates that men are more prone to problematic video gaming than women, while female individuals present a pronounced link with addictive social media consumption [42]. As expected, we found that boys exhibited a higher likelihood of reporting Facebook and/or gaming-related issues, whether these issues were separate or concurrent, compared to girls. Dong et al. elucidated this trend by variances in neural mechanisms linked to gender [43]. In males, exposure to screen practices resulted in increased cravings and demonstrated elevated activity in brain regions, specifically within the corticosteroid-limbic circuitry, associated with reward and an increase in dopamine levels as digital substances with addictive potential [11, 12, 43].

Nonetheless, a recent meta-analysis [44] found that boys demonstrated a higher likelihood of displaying gaming disorder compared to girls. Conversely, boys exhibited a lower likelihood of manifesting social media addiction in contrast to girls. Furthermore, both effect sizes varied across different regions, and were notably greater in Europe and the Americas in comparison to Asia [44]. The high risk of co-occurrence of Problematic Facebook and Video Game Use among boys may be explained not only by biological factors but also by social and behavioral components. Indeed, adolescents use social media to share their video game experiences, including photos, videos, status updates, and links. In return, they receive likes, comments, and reactions which can be reinforcing. This multifaceted phenomenon reflects the engagement of young gamers with gaming culture and their desire for connection, recognition, expression of themselves, and building communities around their shared passion for video games, regardless of geographic distances [45, 46].

Moreover, Facebook hosts various games and entertainment apps, which can be particularly appealing to adolescents. They can play games, participate in quizzes, and engage in other entertainment activities directly on the platform, often connecting and competing with friends. Furthermore, the Messenger app, which was often linked with Facebook, provided a convenient means of communication for adolescents. It allows for real-time chatting, group chats, and the exchange of multimedia content [46]. However, it’s essential to recognize that the popularity of social media platforms can change rapidly due to shifts in trends, evolving demographics, and changes in platform features. In recent years, adolescents have been gradually shifting toward other platforms like Instagram, Snapchat, and TikTok, which offer different experiences [17].

Interestingly, a Norwegian study revealed that boys connected gaming to learning, education, and careers. Several boys envisioned a future where video games would be part of their lives, not solely as a passionate pastime but also as a possible career, such as a professional video gamer (eSports athlete), streamer, or game developer [47].

Notably, our study finding of a correlation between problematic internet use and the co-occurrence of Problematic Facebook and Video Game Use means that adolescents who used heavily the internet were more likely to experience simultaneous digital addictions. In agreement with our research findings, previous studies have endorsed the relationship between the average time spent on the internet and the risk of being Facebook and video game addicted [16, 39, 48, 49]. Błachnio et al. [48] asserted that there is a statistically significant relationship between Problematic Facebook Use and several variables, including gender, age, and daily internet usage. Their findings suggested that increased time spent on the internet, being of a younger age, and identifying as male are all factors linked to elevated levels of Facebook addiction [48]. The relationship between the average daily duration of time spent and digital addictions is possibly accounted for by the linearity hypothesis of the dose/effect curve that makes adolescents simultaneous behavioral addictions. Additional investigation is warranted to fully understand the implications of these findings.

We also considered the impact of mental health disorders on the likelihood of co-occurring Problematic Facebook and Video Game Use. Among adolescents, depression and anxiety emerged as significant predictors of facing problematic use of Facebook and video games. Interestingly, the more severe the depression disorder, the greater the likelihood of co-occurring Problematic Facebook and Video Game Use. Furthermore, individuals with an anxiety disorder had 4.21 times higher odds of experiencing a higher number of addictive behaviors compared to those who did not report anxiety.

Most literature focused on the individual associations between digital addictions and mental health [50]. Yet, we add to the research body the fact that the strength of association is getting higher with the co-occurrence of Problematic Facebook and Video Game Use. This trend is consistent with a study, that was conducted to assess the associations between self-reported alcohol use disorder and mental health problems among young Swiss men, but that the co-occurrence of other behavioral addictions is also associated with increased proportions of mental health problems [51].

Our results are possibly explicable through uses and gratifications theory [2], that is individuals experiencing depression tend to engage in online social communication and/or be spending large amounts of their time engaging in non-social behavior on Facebook, such as playing games to escape negative moods. Consequently, they reinforce their Facebook and video game usage [52]. Additionally, the displaced behavior theory suggests that the more time people spend on social media and playing video games, the less time they allocate to real-world interactions [50]. Adolescents might be dealing with real-world stressors such as academic pressure, family conflicts, or peer problems. Engaging in social media and video games provides a form of escapism, allowing them to temporarily escape these challenges and experience a different reality [53]. Conversely, it remains unclear whether anxiety and depression elevate an adolescent’s risk of developing Problematic Facebook and Video Game Use, or if these addictive behaviors increase the likelihood of anxiety disorders. Thus, warranting comprehensive longitudinal studies that examine the bidirectional relationships between these mental health variables over time.

The study was conducted on a randomly selected group of a large sample size of adolescents using appropriate and reliable research tools. Nonetheless, Results should be interpreted in light of study limitations. The cross-sectional nature of the present study does not allow the results to be interpreted in the context of causality; hence, the study is limited in this regard. However, the study focused only on adolescents in public school, those in private school and out of school were not represented. While our study focused on assessing primary addictive behaviors such as Problematic Facebook Use and Problematic Video Game Use, it is important to note that we did not evaluate gambling, Instagram, or TikTok addiction. These platforms have seen significant spread among adolescents [14], and future research should consider including them in the scope of investigation. An additional potential limitation within our study lies in the utilization of a self-administered questionnaire. This approach carries the risk of introducing reporting bias, which in turn may result in subjectivity that leads to either an overestimation or underestimation of the data. On one hand, certain participants may be inclined to underreport their substance use, influenced by the negative social stigma associated with such behavior in Arab-Muslim societies, particularly among females. On the other hand, some participants might tend to exaggerate their substance use to create a more favorable impression among their peers who were present when they completed the questionnaires.

It also appears essential to properly include a qualitative approach to explore concepts and revelations regarding the behavioral responses of adolescents.

## Conclusion

Problematic Facebook Use and Problematic Video Game Use and its co-occurrence were quite prevalent among a large sample of Tunisian adolescents. The co-occurrence of these addictive behaviors was strongly positively associated with, male gender, problematic internet use, depression disorder, and anxiety disorder. However, it is important to acknowledge that the precise mechanisms underlying these relationships may be more complex. Future research should explore potential mediators like family dynamics, social support, and coping strategies, which may influence how problematic Facebook and video game use relate to mental health issues. Finally, our study highlights the need for a comprehensive, multifaceted approach to address these issues and promote the well-being of our youth in the digital age. The Ministry of Health could incorporate school-based screening for mental health disorders and digital addiction into routine assessments, provide support and resources for affected children, and implement guidelines to promote responsible internet use. Digital literacy programs into the curriculum could be also integrated to teach students about healthy online behaviors coupled with regular awareness campaigns.

### Electronic supplementary material

Below is the link to the electronic supplementary material.

Supplementary Material 1

## Data Availability

No datasets were generated or analysed during the current study.

## Abbreviations

BDI: Beck Depression Inventory
SCARED-C: Screen for Child Anxiety Related Disorders-Child
TAS: Toronto Alexithymia Scale
TND: Tunisian Dinars
AOR: Adjusted Odds Ratio
CI: Confidence Interval

## References

[1] J S, P L. Technological Addictions. Psychiatr Clin North Am. 2022 [cited 2023 Aug 18];45(3). https://pubmed.ncbi.nlm.nih.gov/36055740/.10.1016/j.psc.2022.04.00736055740

[2] Schønning V, Hjetland GJ, Aarø LE, Skogen JC (2020). Social Media Use and Mental Health and Well-being among adolescents – A scoping review. Front Psychol.

[3] Sawyer SM, Azzopardi PS, Wickremarathne D, Patton GC (2018). The age of adolescence. Lancet Child Adolesc Health.

[4] Szwedo DE, Hessel ET, Loeb EL, Hafen CA, Allen JP (2017). Adolescent support seeking as a path to adult functional independence. Dev Psychol.

[5] Goodman A (1990). Addiction: definition and implications. Br J Addict.

[6] Magis-Weinberg L, Ballonoff Suleiman A, Dahl RE (2021). Context, Development, and Digital Media: implications for very young adolescents in LMICs. Front Psychol.

[7] Hasin DS, O’Brien CP, Auriacombe M, Borges G, Bucholz K, Budney A (2013). DSM-5 criteria for Substance Use disorders: recommendations and rationale. Am J Psychiatry.

[8] Rémond JJ, Romo L (2018). Analysis of Gambling in the media related to screens: immersion as a predictor of excessive use?. Int J Environ Res Public Health.

[9] Statista. [cited 2023 Aug 1]. Video Games - Worldwide | Statista Market Forecast. https://www.statista.com/outlook/dmo/digital-media/video-games/worldwide.

[10] Statista. [cited 2023 Aug 20]. Biggest social media platforms 2023. https://www.statista.com/statistics/272014/global-social-networks-ranked-by-number-of-users/.

[11] Kühn S, Romanowski A, Schilling C, Lorenz R, Mörsen C, Seiferth N (2011). The neural basis of video gaming. Transl Psychiatry.

[12] Westbrook A, Ghosh A, van den Bosch R, Määttä JI, Hofmans L, Cools R (2021). Striatal dopamine synthesis capacity reflects smartphone social activity. iScience.

[13] Eliacik K, Bolat N, Koçyiğit C, Kanik A, Selkie E, Yilmaz H (2016). Internet addiction, sleep and health-related life quality among obese individuals: a comparison study of the growing problems in adolescent health. Eat Weight Disord - Stud Anorex Bulim Obes.

[14] Bozzola E, Spina G, Agostiniani R, Barni S, Russo R, Scarpato E (2022). The Use of Social Media in Children and adolescents: scoping review on the potential risks. Int J Environ Res Public Health.

[15] Brailovskaia J, Margraf J (2017). Facebook Addiction Disorder (FAD) among German students-A longitudinal approach. PLoS ONE.

[16] Burleigh TL, Griffiths MD, Sumich A, Stavropoulos V, Kuss DJ (2019). A systematic review of the co-occurrence of Gaming Disorder and other potentially addictive behaviors. Curr Addict Rep.

[17] C C, Yc L, Jw LC. L. Prevalence of social media addiction across 32 nations: Meta-analysis with subgroup analysis of classification schemes and cultural values. Addict Behav. 2021 [cited 2023 Aug 17];117. https://pubmed.ncbi.nlm.nih.gov/33550200/.10.1016/j.addbeh.2021.10684533550200

[18] Faouel N, Soussia RB, Gharbi M, Kacem M, Mohamed AH, Bouali W (2022). Prevalence of Facebook Addiction in a teenage Population: about 110 cases. Eur Psychiatry.

[19] Karim MR, Haque MJ, Akhter S, Ahmed HU (2023). Facebook addiction and its related factors among medical students; a cross- sectional study in Bangladesh. PLOS Glob Public Health.

[20] Khan NT (2018). Facebook Addiction and its Association with academic performance. Biomed J Sci Tech Res.

[21] Benedetti E, Cotichini R, Molinaro S (2022). Adolescent substance use and risk behaviours in the Mediterranean region: fourth MedSPAD regional report.

[22] MedSPAD III 2021 Tunisie: résultats de l’enquête nationale MedSPAD III.pdf. [cited 2024 May 2]. http://www.santetunisie.rns.tn/images/medspad3_2023.pdf.

[23] Patel V, Flisher AJ, Nikapota A, Malhotra S (2008). Promoting child and adolescent mental health in low and middle income countries. J Child Psychol Psychiatry.

[24] Konkolÿ Thege B, Hodgins DC, Wild TC. Co-occurring substance-related and behavioral addiction problems: a person-centered, lay epidemiology approach. J Behav Addict 5(4):614–22.10.1556/2006.5.2016.079PMC537036627829288

[25] Mérelle SYM, Kleiboer AM, Schotanus M, Cluitmans TLM, Waardenburg CM, Kramer D (2017). Which health-related problems are associated with problematic video-gaming or social media use in adolescents? A large-scale cross-sectional study. Clin Neuropsychiatry J Treat Eval.

[26] Li L, Abbey C, Wang H, Zhu A, Shao T, Dai D (2022). The Association between Video Game Time and adolescent Mental Health: evidence from Rural China. Int J Environ Res Public Health.

[27] Shettar M, Karkal R, Kakunje A, Mendonsa RD, Chandran VM (2017). Facebook addiction and loneliness in the post-graduate students of a university in southern India. Int J Soc Psychiatry.

[28] Soua S, Ghammam R, Maatoug J, Zammit N, Ben Fredj S, Martinez F et al. The prevalence of high blood pressure and its determinants among Tunisian adolescents. J Hum Hypertens. 2022;1–9.10.1038/s41371-022-00677-xPMC1100157835396537

[29] Rosenberg M, Schooler C, Schoenbach C, Rosenberg F (1995). Global self-esteem and specific Self-Esteem: different concepts, different outcomes. Am Sociol Rev.

[30] Abdel-Khalek AM (1998). Internal consistency of an arabic adaptation of the Beck Depression Inventory in four arab countries. Psychol Rep.

[31] Beck AT, Rial WY, Rickels K (1974). Short form of depression inventory: cross-validation. Psychol Rep.

[32] Hariz N, Bawab S, Atwi M, Tavitian L, Zeinoun P, Khani M (2013). Reliability and validity of the arabic screen for child anxiety related Emotional disorders (SCARED) in a clinical sample. Psychiatry Res.

[33] Birmaher B, Khetarpal S, Brent D, Cully M, Balach L, Kaufman J (1997). The screen for child anxiety related Emotional disorders (SCARED): scale construction and psychometric characteristics. J Am Acad Child Adolesc Psychiatry.

[34] El Abiddine FZ, Dave H, Aldhafri S, El-Astal S, Hemaid F, Parker JDA (2017). Cross-validation of the 20-item Toronto Alexithymia Scale: results from an arabic multicenter study. Personal Individ Differ.

[35] Loas G, Braun S, Delhaye M, Linkowski P (2017). The measurement of alexithymia in children and adolescents: psychometric properties of the Alexithymia Questionnaire for Children and the twenty-item Toronto Alexithymia Scale in different non-clinical and clinical samples of children and adolescents. PLoS ONE.

[36] Parker JDA, Taylor GJ, Bagby RM (2003). The 20-Item Toronto Alexithymia Scale. III. Reliability and factorial validity in a community population. J Psychosom Res.

[37] Ghali H, Ghammem R, Zammit N, Fredj SB, Ammari F, Maatoug J et al. Validation of the arabic version of the Bergen Facebook Addiction Scale in Tunisian adolescents. Int J Adolesc Med Health. 2019;34(1).10.1515/ijamh-2019-007731550234

[38] Messedi N, Chakroun M, Smaoui N, Halouani N, Ellouze S, Turki M et al. L’Addiction au reseau social facebook chez les etudiants en medecine.

[39] Cherif L, Ayadi H, Khmakhem K, Kacem IH, Kammoun S, Moalla Y. Problematic Video Game Use among Teenagers in Sfax, Tunisia. J Health Educ Res Dev. 2018 [cited 2023 Aug 17];06(03). https://www.omicsonline.org/open-access/problematic-video-game-use-among-teenagers-in-sfax-tunisia-2380-5439-1000268-104046.html.

[40] Sherer J, Levounis P (2022). Technological addictions. Psychiatr Clin North Am.

[41] Potas N, Açıkalın ŞN, Erçetin ŞŞ, Koçtürk N, Neyişci N, Çevik MS (2022). Technology addiction of adolescents in the COVID-19 era: mediating effect of attitude on awareness and behavior. Curr Psychol N B Nj.

[42] Andreassen CS, Billieux J, Griffiths MD, Kuss DJ, Demetrovics Z, Mazzoni E (2016). The relationship between addictive use of social media and video games and symptoms of psychiatric disorders: a large-scale cross-sectional study. Psychol Addict Behav.

[43] Dong G, Wang L, Du X, Potenza MN (2018). Gender-related differences in neural responses to gaming cues before and after gaming: implications for gender-specific vulnerabilities to internet gaming disorder. Soc Cogn Affect Neurosci.

[44] Su W, Han X, Yu H, Wu Y, Potenza MN (2020). Do men become addicted to internet gaming and women to social media? A meta-analysis examining gender-related differences in specific internet addiction. Comput Hum Behav.

[45] Kowert R, Domahidi E, Quandt T (2014). The relationship between online video game involvement and gaming-related friendships among emotionally sensitive individuals. Cyberpsychology Behav Soc Netw.

[46] Nadkarni A, Hofmann SG (2012). Why do People Use Facebook?. Personal Individ Differ.

[47] Leonhardt M, Overå S (2021). Are there differences in Video Gaming and Use of Social Media among boys and girls?—A mixed methods Approach. Int J Environ Res Public Health.

[48] Błachnio A, Przepiórka A, Pantic I (2015). Internet use, Facebook intrusion, and depression: results of a cross-sectional study. Eur Psychiatry J Assoc Eur Psychiatr.

[49] Khumsri J, Yingyeun R, Mereerat Manwong null, Hanprathet N, Phanasathit M. Prevalence of Facebook Addiction and Related Factors Among Thai High School Students. J Med Assoc Thail Chotmaihet Thangphaet. 2015;98 Suppl 3:S51-60.26387389

[50] Karim F, Oyewande AA, Abdalla LF, Chaudhry Ehsanullah R, Khan S. Social Media Use and its connection to Mental Health: a systematic review. Cureus 12(6):e8627.10.7759/cureus.8627PMC736439332685296

[51] Marmet S, Studer J, Lemoine M, Grazioli VS, Bertholet N, Gmel G (2019). Reconsidering the associations between self-reported alcohol use disorder and mental health problems in the light of co-occurring addictions in young Swiss men. PLoS ONE.

[52] Ryan T, Xenos S (2011). Who uses Facebook? An investigation into the relationship between the Big Five, shyness, narcissism, loneliness, and Facebook usage. Comput Hum Behav.

[53] Yen JY, Yen CF, Chen CS, Wang PW, Chang YH, Ko CH (2012). Social anxiety in Online and Real-Life Interaction and their Associated factors. Cyberpsychology Behav Soc Netw.

